# Genome-Wide Association Analysis Identifies a Mutation in the Thiamine Transporter 2 *(SLC19A3)* Gene Associated with Alaskan Husky Encephalopathy

**DOI:** 10.1371/journal.pone.0057195

**Published:** 2013-03-04

**Authors:** Karen M. Vernau, Jonathan A. Runstadler, Emily A. Brown, Jessie M. Cameron, Heather J. Huson, Robert J. Higgins, Cameron Ackerley, Beverly K. Sturges, Peter J. Dickinson, Birgit Puschner, Cecilia Giulivi, G. Diane Shelton, Brian H. Robinson, Salvatore DiMauro, Andrew W. Bollen, Danika L. Bannasch

**Affiliations:** 1 University of California Davis, Davis, California, United States of America; 2 University of Alaska Fairbanks, Fairbanks, Alaska, United States of America; 3 Research Institute, The Hospital for Sick Children, Toronto, Ontario, Canada; 4 Department of Pathology, University of California San Diego, La Jolla, California, United States of America; 5 Department of Neurology, Columbia University Medical Center, New York, New York, United States of America; 6 Department of Pathology, School of Medicine, University of California San Francisco, San Francisco, California, United States of America; Utrecht University, The Netherlands

## Abstract

Alaskan Husky Encephalopathy (AHE) has been previously proposed as a mitochondrial encephalopathy based on neuropathological similarities with human Leigh Syndrome (LS). We studied 11 Alaskan Husky dogs with AHE, but found no abnormalities in respiratory chain enzyme activities in muscle and liver, or mutations in mitochondrial or nuclear genes that cause LS in people. A genome wide association study was performed using eight of the affected dogs and 20 related but unaffected control AHs using the Illumina canine HD array. *SLC19A3* was identified as a positional candidate gene. This gene controls the uptake of thiamine in the CNS via expression of the thiamine transporter protein THTR2. Dogs have two copies of this gene located within the candidate interval (*SLC19A3.2* – 43.36–43.38 Mb and *SLC19A3.1* – 43.411–43.419 Mb) on chromosome 25. Expression analysis in a normal dog revealed that one of the paralogs, *SLC19A3.1*, was expressed in the brain and spinal cord while the other was not. Subsequent exon sequencing of *SLC19A3.1* revealed a 4bp insertion and SNP in the second exon that is predicted to result in a functional protein truncation of 279 amino acids (c.624 insTTGC, c.625 C>A). All dogs with AHE were homozygous for this mutation, 15/41 healthy AH control dogs were heterozygous carriers while 26/41 normal healthy AH dogs were wild type. Furthermore, this mutation was not detected in another 187 dogs of different breeds. These results suggest that this mutation in *SLC19A3.1,* encoding a thiamine transporter protein, plays a critical role in the pathogenesis of AHE.

## Introduction

Alaskan Husky Encephalopathy (AHE) is a fatal brain disease in young Alaskan Husky (AH) dogs, often affecting multiple dogs from the same litter [1], [2]. AHE was initially described in 13 dogs from the northern United States, including Alaska, Massachusetts, New York, Wyoming, Maine and Minnesota [1]. Based on the clinical and neuropathological similarities to Leigh Syndrome (LS) in people, AHE was proposed to be a mitochondrial encephalopathy. Human LS includes a group of diseases with heterogeneous clinical symptoms, usually characterized by elevations in blood lactate and respiratory chain enzyme dysfunction(s), and due to various mutations in either nuclear or mitochondrial DNA. An almost identical clinicopathological disease to AHE is described in 11 European Yorkshire terriers without a defined underlying cause [3].

Dogs with AHE may have acute onset of clinical signs, or chronic progressive waxing and waning clinical history. Typically, they have multifocal central nervous system deficits including seizures, altered mentation, dysphagia, absent menace response, central blindness, hypermetria, proprioceptive positioning deficits, facial hypoalgesia, ataxia and tetraparesis.

Diagnostic testing reported in dogs with AHE was limited to normal serum and cerebrospinal fluid pyruvate and lactate concentrations; evaluation of mitochondrial respiratory chain enzymes was not done. Two dogs also had intracranial imaging. Computed tomography images in one dog had bilateral hypoattenuating lesions in the thalamus, and MR images of the other dog had bilateral hyperintense lesions in the brainstem on T2 weighted images. All dogs died or were euthanized, most within 2–7 months, however one dog lived for 1 year after the onset of clinical signs when it died of “natural causes” [1], [2].

In people and domestic animals, a multitude of uncommon diseases are associated with bilateral and symmetrically distributed brain lesions, apparent on magnetic resonance imaging and/or neuropathology. Examples include toxicities (carbon monoxide poisoning), metabolic (Leigh Syndrome [4], hypoxic-ischemic encephalopathy, hypoglycemia, biotin responsive basal ganglia disease [5], Wernicke's-like encephalopathy [6]), inflammatory (Neuro Behcet disease), nutritional (thiamine deficiency encephalopathy [7]), vascular (deep cerebral vein thrombosis), infectious (bovine spongiform encephalopathy, Creutzfeld-Jakob disease), and inborn errors of metabolism (L-2 hydoxyglutamic aciduria [8], citrullinemia). A systematic diagnostic approach to this group of disorders is essential to ensure that a specific diagnosis can be rendered in a timely manner.

In people, mutations in the *SLC19A3* gene (encoding a thiamine transporter protein) are associated with encephalopathies that have some clinical and neuropathologic similarities to AHE [9]. In this study, 11 dogs with neuropathologically and/or neuroradiologically confirmed AHE were evaluated for 1) mitochondrial respiratory chain enzyme functions; 2) light and electron microscopical pathological studies on skeletal muscle and liver, and 3) a genome wide association study utilizing the Illumina canine HD array. Together, our findings suggest that the pathogenesis of AHE results from a genetic defect in a thiamine transporter (*SLC19A3*), and is not a primary mitochondrial encephalopathy.

## Results

### Clinical Findings and Outcome in dogs with AHE

All 11 dogs with AHE included in this study showed typical clinical signs (**Table** **1**), as well as MR imaging **(** **Figure** **1** **)** and/or neuropathological features of AHE in the brain **(** **Figure** **2** **).** Of these 11 dogs, 6 were euthanized either immediately after their clinical evaluation (dogs # 1, 3, 6, 8, 9, 11), or six months (dog #5) or 27 months later (dog #2) **(** **Table** **1**). Parents of each of the affected dogs were clinically normal. Three sets of 2 dogs were littermates. Dog #9 whelped a litter of clinically normal puppies (6 puppies), 8 months prior to developing clinical signs of AHE.

**Figure 1:** (upper panel). MRI images (T2-weighted, transverse) of a normal brain from a clinically normal 1 year old male Alaskan Husky (C#1). **Figure** **1** **and** **2** **a** are at the level of the head of the caudal nucleus, **Figure** **1** **and** **2** **b** are at the level of the temporomandibular joint, and **Figure** **1** **and** **2** **c** are at the level of the bulla. **Lower panel:** MR images (T2 weighted, transverse) from the brain of dog #3 with neuropathologically confirmed AHE. There are multifocal regions of abnormal hyperintensity in the brain, which are bilateral and symmetrical (arrows). **a.** Hyperintense lesions are present in the lateral aspect of the caudate nucleus, claustrum and putamen. **b.** Bilaterally symmetrical lesions in the thalamus and at the base of the sulci, at the junctional grey and white matter in the cerebral hemispheres. **c.** Hyperintense lesions in the medulla, vermis of the cerebellum, and in the cerebrum.

**Figure 2:** Brain of dog #6. **A**. Transverse section of brain with bilaterally symmetrical areas of cavitation due to encephalomalacia in the thalamus. **B.** Same dog; macrophotograph of a transverse section of brain rostral to Figure 2A illustrating bilaterally symmetrical areas of polioencephalomalacia [2] or of necrosis with incipient malacia [1], [3], [4] in cortex deep in the sulci [1], in the claustrum [2], in caudate nucleus [3] and the globus pallidus [4] (HE-LFB stain).

**Table 1:** Signalment, Presenting Clinical Signs, and Long Term Outcome of Alaskan Huskies with AHE.

Dog #	Sex	Age at presentation (months)	Seizures	Tetraparesis	Generalized Ataxia	Thoracic Limb Hyper-metria	Dysphagia	Central Blindness	Longterm Outcome
1	F	8	Y	N	Y	Y	N	N	Euthanized
2	M	8	Y	Y	Y	Y	N	N	Euthanized 27 months post diagnosis
3	F	12	N	Y	Y	N	Y	Y	Euthanized
4	F	6	Y	Y	Y	Y	N	N	Alive
5	M	6	Y	Y	Y	Y	N	N	Euthanized 6 months post diagnosis
6	F	8	N	Y	Y	N	Y	Y	Euthanized
7	F	21	N	Y	Y	N	Y	N	Alive 27 months post diagnosis
8	M	9	Y	Y	Y	N	N	N	Euthanized
9	F	24	Y	N	N	N	N	N	Euthanized
10	M	8	N	N	Y	Y	Y	N	Alive 7 months post diagnosis
11	M	6	Y	Y	Y	N	N	N	Euthanized

Dog #2 clinically improved and was neurologically stable 6 months after presentation. He had mild neurological deficits consisting of proprioceptive placing deficits in all four limbs, and infrequent generalized seizures. Clinical signs were static for the next 21 months, followed by a rapid progression. A repeat MRI showed increased size of the previously defined lesions. The dog was euthanized 27 months after presentation. Dog #4 is alive 51 months after initial presentation with continuing but static neurological deficits. An MRI was repeated 12 months after the initial MRI, and no changes were noted. Dog #5 had static neurological deficits for 5 months after presentation, but then developed progressive clinical signs, and was euthanized one month later. Repeat MRI 4 months after the initial one demonstrated increased size of the previously noted lesions. Dog #7 is alive with static neurological deficits 32 months after diagnosis; Dog #10 is alive 12 months after initial presentation. However seizures, worsening ataxia and hypermetria developed 4 months after being hit by a car and fracturing the pelvis. The neurological deficits have been static for the previous 9 months.

### Control Alaskan Husky dogs

One normal AH dog with a normal physical, neurological examination and brain MRI evaluation was admitted into this study (C#1). Blood samples from 41 apparently healthy normal AH dogs from three racing kennels were obtained for genotyping.

### Control non-Alaskan Husky dogs

Blood samples for genotyping were obtained from 187 randomly chosen canine patients from the VMTH including 51 breeds of both sexes and of varying ages, with a broad spectrum of clinical diseases. A skin biopsy sample for fibroblast culture was obtained from one dog with intervertebral disc disease at the time of laminectomy. Muscle biopsies were collected from one dog with a fractured femur (from the non-fracture leg) immediately after euthanasia.

### Mitochondrial respiratory chain enzyme assays

Respiratory chain enzyme activities were measured in mitochondria from liver **(** **Table** **2** **)** and skeletal muscle homogenates **(** **Table** **3** **).** There were no major differences between the activities in the AHE and control dogs either before or after standardization with citrate synthase and succinate dehydrogenase. Likewise, pyruvate dehydrogenase complex and 2-14C whole cell oxidation measurements were normal (data not shown).

**Table 2:** Respiratory chain enzyme rates in liver of dogs with AHE.

Dog #	CI+III* (nmol/mg/min)	CI+III/CS	CII+III (nmol/mg/min)	CII+III/CS	CIV (nmol/mg/min)	CS (nmol/mg/min)	CIV/CS
C#1	1.53	0.30	4.64	0.90	10.81	5.15	2.10
1	2.27	0.51	3.24	0.74	14.20	4.41	3.22
3	2.02	0.47	1.00	0.23	4.55	4.27	1.07
4	1.34	0.36	1.58	0.42	7.68	3.73	2.06
5	1.54	0.29	1.98	0.37	12.60	5.35	2.36

* CI+III (complex I+III), NADH: cytochrome c reductase; CII+III (complex II+III), succinate:cytochrome c reductase; CIV (complex IV), cytochrome oxidase; CS (citrate synthase).

**Table 3:** Respiratory chain enzyme rates in skeletal muscle of dogs with AHE.

Complex	Dog #1	Dog #2	Dog #2 (repeat)	Control non AH Dog
I+III	1.05	1.01	3.45	0.72
I	31.74	30.66	35.91	28.52
II+III	0.74	0.73	0.91	0.32
IV	2.66	2.65	3.23	2.30
SDH	1.41	1.15	1.77	0.64
CS	40.43	31.29	34.96	33.70
Values/CS				
I+III	0.026	0.032	0.098	0.021
I	0.79	0.98	1.03	0.85
II+III	0.018	0.023	0.026	0.0094
IV	0.066	0.085	0.092	0.068
SDH	0.035	0.037	0.051	0.019
Values/SDH				
I+III	0.74	0.88	1.95	1.12
I	22.51	26.7	20.20	52.66
II+III	0.52	0.63	0.51	0.50
IV	1.89	2.30	1.82	3.59
CS	28.67	27.2	19.75	52.7

* SDH  =  succinate:dehydrogenase; CS  =  citrate synthase.

### Biochemical assays in blood and cerebrospinal fluid (CSF)

No abnormalities were noted on the CBC, CSF and serum biochemistry analysis in any dog. There was no indication of a mitochondrial disorder on evaluation of plasma or CSF lactate or pyruvate levels, or in the lactate to pyruvate ratios.

### Neuropathology findings

Seven dogs were euthanized and 5 had a necropsy. In 2 dogs, only the brain was evaluated pathologically. All dogs had neuropathological lesions characteristic for AHE with minor differences in severity among dogs, but not in location. In all dogs, bilaterally symmetrical areas of cystic encephalomalacia were grossly visible in the thalamus **(** **Figure** **2A** **).** Microscopically, lesions also included foci of bilaterally symmetrical polioencephalomalacia in the claustrum (**Figure** **2B** **(1))**, or of necrosis with incipient malacia (in the deep gray and underlying white matter of the cerebral cortex confined to the base of the sulci **(** **Figure** **2B** **(1)**, in the claustrum **(** **Figure** **2B** **(2)**, putamen, caudate nucleus **(** **Figure 2B** **(3),** globus pallidus **(** **Figure 2B** **(4)**, pons, and medulla oblongata. There were similar but milder bilaterally symmetrical malacic lesions in the deep in the midline of the ventral lobes of the vermis.

Frozen fresh muscle was histochemically stained and evaluated by light microscopy in 2 dogs with AHE. In one dog (dog #1) the muscle was normal. In the other more severely affected dog (dog #2), deposits of succinic dehydrogenase (**Figure** **3**) and cytochrome *c* oxidase positive material were noted, most consistent with mild mitochondrial proliferation. Ultrastructural lesions in the skeletal muscle from two affected dogs (dogs #4 and #5) were compared with one normal AH dog (C#1) (Muscle from dogs #1 and #2 was not evaluated ultrastructurally. Muscle from dogs #4 and #5 was not evaluated by light microscopy). In both dogs #4 and #5, enlarged megamitochondria (2–9 μm diameter, compared to the control dog C#1, where the diameter was 0.5 μm) were observed with the novel finding of abnormal glycogen deposits inside the mitochondria. Ultrastructurally, glycogen accumulation was also found in large aggregates outside the mitochondria. The mitochondrial cristae were disorganized with whorls **(** **Figure** **4** **)**.

**Figure 3:** Frozen muscle section from dog #2, histochemically stained with succinic dehydrogenase (SDH). There are areas of excessive SDH positive staining (arrow) in two myofibers, most consistent with mild mitochondrial proliferation.

**Figure 4:** Fixed muscle (dog #4). Transmission electron microscopy. Glycogen deposits (arrowhead) are present in the abnormal megamitochondria (arrow).

### Molecular Genetic Studies

Many of the mitochondrial DNA candidates for human Leigh Syndrome were sequenced in affected dogs (MT-ATP8/6, MT-tRNA^LYS^, MT-tRNA^LEU(UUR)^, MT-tRNA^SER(AGY)^, MT-tRNA^TRY^, MT-tRNA^TYR^, MT-tRNA^VAL^) with no mutations identified in one of either blood, liver or fibroblast DNA.

In addition, the following genes were also sequenced: *POLG*, *Twinkle*, *DGUOK*, *RRMB2*, *MPV17*, *SUCLA2*, *SUCLG1*, *TK2*. Depending on the gene, either gDNA or cDNA from fibroblasts were sequenced; no mutations were identified in any gene.

### Genome Wide Association Study

Whole genome association was performed using 8 AHE affected dogs (dogs #1–8) and 20 unaffected but related controls. The genomic inflation factor for this group of samples was 1 indicating that there was little population stratification. After pruning, 114,613 SNPs were available for analysis. Raw p values showed a cluster of SNPs located on CFA (*Canis familiaris*) 25 with values 56 times lower than for the next best associated SNP on CFA 30. Permutation testing did not give genome wide significance for the best associated SNPs, however the strong signal from many SNPs from one discrete location and the absence of any signal from other chromosomes warranted further investigation. When genotypes from this area were analyzed, a region of complete homozygosity was identified in all the affected dogs and never in the 20 unaffected dogs. The region of homozygosity extended 3.5 Mb between 41074763 and 44542154 (**Figure** **5**).

**Figure 5:** Genome wide association analysis of Alaskan Husky encephalopathy. A. Manhattan plot of –log 10 of raw p values (y axis) by chromosome (x axis). The best associated SNP (p = 6.59×10^−6^) was located at 43980115 Mb on Cfa 25 B. –log 10 of the permuted (100,000)p values (y axis) are plotted by chromosome (x axis). The lowest p value (0.051) was obtained for the same SNP located at 43980115 Mb. C. The Chi square value shown in grey and the allele frequency shown in black on the y axis are plotted against the Mb (x axis) on CFA 25. The location of the two paralogs of *SLC19A3* are shown within the region of homozygosity identified in the affected individuals at the top of the figure.

### *SLC19A3* Expression

Evaluation of this region for candidate genes uncovered SLC19A3 as a likely candidate, based on the phenotypic similarities between people affected with biotin-responsive basal ganglia disease (BBGD) and dogs with AHE. In the canine genome there has been a duplication of *SLC19A3* and there are two paralogs, *SLC19A3.1* (43,411,960–43,419,612 Mb) and *SLC19A3.2* (43,363,905–43,386,983 Mb). *SLC19A3.1* shares 84.7% identity and *SLC19A3.2* shares 79.9% identity at the amino acid level with the human gene. In order to determine which gene was the more likely candidate, the tissue specific expression levels of each gene were evaluated **(** **Figure** **6** **)**. *SLC19A3.1* was expressed in the cerebrum, cerebellum and spinal cord while *SLC19A3.2* was not. In addition, *SLC19A3.1* had higher nucleotide homology to the human locus, therefore it was pursued as the best regional candidate gene.

**Figure 6:** The relative tissue specific expression levels of the two paralogs of *SLC19A3* and GAPDH. RT PCR products obtained from equal amounts of cDNA are shown from the following tissues: 1 spleen, 2 skin, 3 cerebellum, 4 thymus, 5 testis, 6 spinal cord, 7 heart, 8 muscle, 9 cerebral cortex, 10 kidney, and 11 liver.

### *SLC19A3* Sequencing

The coding region of *SLC19A3.1* was sequenced as well as some intronic sequences. Four changes were identified in dogs with AHE relative to both the canfam2 Boxer sequence and an unaffected AH control (**Table** **4**). A 4 bp insertion (c.624 insTTGC) and SNP (c.625 C>A) in exon 2 were the most compelling changes since they were predicted to result in a frame shift and premature peptide termination which would truncate 279 amino acids of the 498 amino acid full length protein (**Figure** **7**). In order to test additional animals, a genotyping assay based on PCR product size was developed for this insertion. All 11 dogs with AHE were homozygous for the mutation, 26/41 unaffected AH dogs were homozygous wild type and 15/41 unaffected AH dogs were determined to be heterozygous carriers. In order to determine if the deletion was just a polymorphism, 187 dogs from 51 breeds were genotyped and the mutant allele was not identified. Expression levels of *SLC19A3.1* were compared in cerebral cortex tissue from a dog affected with AHE and an unaffected beagle sample and *SLC19A3.1* expression was dramatically decreased in the affected dog (**Figure** **8**)**.**

**Figure 7:** DNA sequence of the mutation identified in AHE. A. wildtype sequence, B. Heterozygous carrier, C. Mutant sequence.

**Figure 8:** The relative expression levels of *SLC19A3.1* in canine cerebral cortex. RT PCR from equal amounts of RNA isolated from a normal beagle and an Alaskan husky sled dog affected with AHE.

**Table 4:** Sequencing results of *SLC19A3* in dogs with AHE.

Mutation	Location	Change in DNA (5′ to 3′)	Change in Protein
12 bp insertion intron 1	chr25:43,417,532 [191 bp downstream from ex2 (chr25:43,417,341)]	CTTTCTTTCTTT	none
SNP 1 exon 2	chr25:43,417,105	C>T	none
SNP 2 exon 2 + 4 bp insertion	chr25:43,416,868	G>T + TTGC	Amino Acid 208: Gln>His, out of frame for 10 AA, protein termination at AA 219
8 bp deletion intron 2	chr25:43,414,774-43,414,781 [79 bp downstream ex 3 (chr25:43,414,702)]	AAATAAAT	none
SNP exon 5	chr25:43,411,974	A>G	Amino Acid 490: Thr>Ala

## Discussion

We have demonstrated in this study that a homozygous mutation in the *SLC19A3.1* gene encoding a thiamine transport protein is strongly associated with AHE. Each of the 11 dogs with AHE had a homozygous mutation of *SLC19A3.1*, and 15/41 clinically normal AH dogs had a heterozygous mutation while the other 26 had wild type homozygosity. No such mutation was found in any of the 187 non-AH dog breeds. Although AHE has been claimed to be a primary mitochondrial encephalopathy based on clinical and pathological similarities to LS, no mutations were found in any of the candidate canine nuclear or mitochondrial genes linked to human LS. In dogs with AHE, biochemical analysis failed to demonstrate defects in the mitochondrial respiratory chain enzyme activities in liver, skeletal muscle or cultured fibroblasts, considered characteristic of LS. Together, these findings strongly suggest that the pathogenesis of AHE involves a primary defect in a thiamine transporter protein in the CNS and is not due to a primary mitochondrial encephalopathy. However, the AHE phenotype is consistent with a secondary mitochondrial disease.

Solute carrier family 19 (*SLC19*) is a group of genes that transport water-soluble vitamins into cells. [10] There are 3 members in the family, *SLC19A1, SLC19A2* and *SLC19A3*. The *SLC19A1* gene encodes folate transporter 1 protein, regulating intracellular levels of folate, as well as mediating methotrexate transport. The *SLC19A2* gene encodes the human thiamine transporter 1 (hTHTR1) protein whereas human thiamine transporter 2 (hTHTR2) protein is encoded by the *SLC19A3* gene. *SLC19A2* and *SLC19A3* are structurally and functionally similar and thiamin (vitamin B1) is transported across the cell membrane by both thiamine transporters. All *SLC19* family genes are expressed ubiquitously, although at variable levels in different tissues [10]. The dog is unusual in that it has two *SLC19A3* paralogs, compared with only one each in mice and people [11]. In the dog, expression of *SLC19A3* is also ubiquitously distributed, but the relative tissue expression varies depending on the specific paralog. In this study, we demonstrated that the CNS has high tissue expression of the *SLC19A3.1* compared with *SLC19A3.2* with *SLC19A3.2* expressed at low levels in the CNS. This finding suggests that *SLC19A3.2* in the CNS cannot compensate for a functional loss of thiamine transport caused by the defective *SLC19A3.1*. In people, *SLC19A3* is expressed at high levels in kidney, liver and placenta, with low levels in other tissues, including the brain [12]. The highest level of *SLC19A3* RNA expression in the human brain is in the thalamus [6]. If the same holds true in the dog, the need for relatively high *SLC19A3* RNA expression in the thalamus could explain the location of the most severe lesions in dogs with AHE [2].

Thiamine is an essential nutrient and thiamine deficiency (TD) may cause bilaterally symmetrical brain lesions in domestic animals and people [7], [13], [14]. Thiamine, a B-complex, water-soluble essential vitamin, has a fundamental role in carbohydrate metabolism in all cells and a critical role in mitochondrial metabolism [15], [16]. Because of the critical dependence of the CNS on mitochondria for energy metabolism, TD can lead rapidly to severe neurological deficits. In dogs, the classical histological lesion of TD (both experimental and spontaneous) is bilaterally symmetrical polioencephalomalacia, confined to the brain stem nuclei, periventricular grey matter, claustrum, lateral geniculate nuclei, caudal colliculi, occipital and parietal cortex, and cerebellar nodulus. Lesions in the caudal colliculus are the hallmark of dietary thiamine deficiency encephalopathy in dogs. Dogs with experimental TD also have cardiac lesions [7]. The distribution of these lesions in the dog differs from those in people, in whom the mammillary bodies are mainly affected, and involvement of the cerebral cortex is more pronounced.

While dogs with TD and AHE have the same histological lesions of bilaterally symmetrical encephalomalacia, anatomic patterns of lesion distribution are distinctively different. Dogs with AHE do not have lesions in the caudal colliculus or lateral geniculate nucleus, and dogs with TD do not have thalamic lesions [2], [7]. In people with spontaneous TD (Wernicke's encephalopathy) who are still responsive to thiamine administration, the lesions are mainly confined to the mammillary bodies. While it is unlikely that the pathogenesis of AHE is due to an absolute global TD, these findings may be consistent with a localized TD, resulting from the functional mutations apparently restricted to the tissue distribution of the *SLC19A3.1* gene.

There is a phenotypic spectrum of diseases in people associated with abnormalities in different regions of the *SLC19A3* gene, including biotin-responsive basal ganglia disease (BBGD) [17], Wernicke's-like encephalopathy (WLE)[6], and an encephalopathy described in 4 related Japanese boys [9]. People with BBGD have vague clinical signs including confusion and vomiting, progressive loss of motor function, dysarthria, dysphagia, cogwheel rigidity, and seizures, which are ultimately fatal if untreated. The major features on brain MRI are areas of bilaterally symmetrical polioencephalomalacia of the caudate and putamen nuclei [17]. Two homozygous missense mutations (c.68G>T; p.G23V; and c.1264A>G, p.T422A) in *SLC19A3* have been identified. In patients with either mutation, no clinical response is noted following thiamine administration. However, if treated with biotin early in the course of disease, the clinical signs may be reversed [17]. In two adult siblings with BBGD, two heterozygous mutations in *SLC19A3* (c.74dupT/p.Ser26LeufsX19 and c.980-14 A>G) led to a premature termination codon (PTC), and a loss of function mutation of *SLC19A3*. One patient responded to biotin, but the other did not improve with biotin administration until thiamine was concurrently supplemented.[18] However, since hTHTR2 does not transport biotin, both the pathophysiology of BBGD, and the response to therapy with biotin imply that a more complex mechanism than simple thiamine deficiency causes these lesions [19]. For example, perhaps the truncated form of the transporter is still able to transport biotin albeit not to the same level as the wild type form, or perhaps since biotin is an important cofactor of many carboxylases in mitochondria, biotin supplementation may exert a compensatory effect.

WLE was reported in 2 Japanese brothers in their second decade of life. Clinical signs included diplopia, external ophthalmoplegia, ptosis, seizures, nystagmus and ataxia. On brain MRI there were hyperintensities on the FLAIR (fluid attenuated inversion recovery) sequences bilaterally in the thalamus and periaqueductal region, which are entirely consistent with actual Wernicke's encephalopathy (thiamine deficiency encephalopathy). A compound heterozygous mutation of p.K44E and p.E320Q was found in *SLC19A3*, resulting in approximately 60% thiamine intracellular uptake in Chinese hamster cells transfected with constructs containing either p.K44E or p.E320Q cDNA compared to the wild-type. Neither patient had serum thiamine deficiency, but both patients responded clinically to thiamine [6].

In four related Japanese boys with infantile seizures, psychomotor retardation, and characteristic lesions on brain MRI (focal T2W hyperintensity in bilateral symmetrical thalamic and basal nuclei, with cerebellar and cerebral cortical atrophy), a homozygous mutation was found (c.958G>C, p.E320Q) in *SLC19A3.* There was no change in either neurological symptoms or brain MRI lesions in response to biotin administration in the one boy who was treated [9].

In BBGD, WLE, and in the Japanese boy encephalopathy, there is a distinct genotype-phenotype correlation. Patients affected by each disease have a remarkably similar phenotype. While the BBGD phenotype is thought to be secondary to a loss-of-function mutation, the Japanese boy encephalopathy may be due to a toxic gain-of-function secondary to the *SLC19A3* mutation [9]. Further investigations are needed to characterize the function effects of these *SLC19A3* mutations and the associated genotypic-phenotypic correlation.

Dogs with AHE did not have any biochemical evidence of primary mitochondrial disease in liver, skeletal muscle or fibroblasts, but did have subtle evidence of mitochondrial pathology. By light microscopy, there was prominent mitochondrial hyperplasia in muscle and liver and ultrastructural examination of muscle revealed “megamitochondria” and abnormal glycogen deposits. However such abnormal mitochondrial morphology is not necessarily evidence of a primary mitochondrial disease. The observed mitochondrial changes could be epiphenomenal, reflective of a response to a defect in energy metabolic pathways as expected with a defective *SLC19A3* gene, especially in an active racing breed.

In conclusion, we have demonstrated that a homozygous mutation in *SLC19A3.1,* a gene encoding a thiamine transport protein in the brain, is strongly associated with AHE. The mutation is homozygous in dogs with AHE while unaffected AH are either homozygous wild type or heterozygous for the mutation. While our findings are consistent with the mutation identified being widespread in AH from North America, we do not know to what extent this or similar mutations might be causal to AHE worldwide. We are hopeful that the findings from this study will help in future studies to test for this mutation in AH from Europe and other regions of the world. While the pathologic findings in AHE are not consistent with classical experimental or spontaneous global TD, they may be consistent with localized TD or may suggest more complex pathways involved with thiamine metabolism in the CNS. This large animal model may allow for prospective investigations into the mechanisms of *SLC19A3* related syndromes and the potential role of thiamine and/or biotin as a therapeutic strategy.

## Materials and Methods

### Criteria for inclusion into the study

#### a. Alaskan Husky dogs with AHE

Alaskan Husky dogs with clinical signs suggestive of AHE, including generalized seizures, gait abnormalities, dysphagia and ataxia [1] (see **Table** **1**), were examined at the VMTH. Dogs had physical and neurological examinations completed by one author, a board certified veterinary neurologist (KV). Dogs that were subsequently euthanized had an immediate necropsy evaluation. For dogs not clinically evaluated at the VMTH, brain MR images were reviewed by four authors (KV, PD, BS and RJH), and/or the formalin fixed brain examined neuropathologically by a board certified veterinary pathologist (RH) and a human neuropathologist(AWB). Neuroimaging and neuropathological lesions that were inclusion criteria for dogs with AHE included bilaterally symmetrical, cavitatory malacic lesions in the thalamus, and smaller malacic lesions in the putamen, claustrum, junctional grey and white matter in the cerebral cortex, in the brainstem and midline cerebellar vermis **(** **Figure** **1** **,** **2A and 2B**). [**2**] All lesions were hyperintense on T2W MR images.

#### b. Control Alaskan Husky dogs

Inclusion criteria for the one healthy, negative control AH was an age greater than one year of age, normal physical and neurological examination, and normal MRI of the brain with no detectable lesions in T1-weighted (T1W) pre- and post contrast, T2-weighted (T2W), proton density weighted, and FLAIR images in both the transverse and sagittal planes. Inclusion criteria for the other dogs were that they were reportedly healthy, older than one year of age, actively racing AHs of both sexes.

#### c. Control non-Alaskan Husky dogs

Non-Alaskan Husky control dogs were randomly selected from canine patients of both sexes and of varying ages admitted to the VMTH during the study period. These control dogs had a wide range of clinical diseases such as kidney disease and intervertebral disc disease, but none had similar clinical signs to AHE. All studies were done with their owner's consent, and in strict accordance with good animal practice, with study protocols approved by the Institutional Animal Care and Use Committee (IACUC) at UC Davis.

### Tissue Culture

Skin biopsies were obtained and fibroblasts were grown and maintained in Eagle's minimal essential medium culture medium, containing 2 mM glutamine (Invitrogen, Burlington, ON, Canada), 1% penicillin/streptomycin and 20% fetal calf serum (Wisent, St-Bruno, Quebec, Canada).

### Mitochondrial Respiratory Chain Enzyme Assays in Skeletal Muscle, Liver and Cultured Fibroblasts

Skeletal muscle and liver specimens were collected under general anesthesia or at necropsy and immediately frozen. Enzyme activities in both skeletal muscle and liver samples were assayed for NADH:cytochrome *c* reductase (Complex I+III), citrate synthase activity, succinate cytochrome *c* reductase (complex II+III) [20], cytochrome oxidase (complex IV) [21] and standardized with respect to citrate synthase and succinate dehydrogenase. 2-^14^C pyruvate whole cell oxidation was measured from cultured fibroblasts as previously described [22] and total pyruvate dehydrogenase complex activity was measured in both the native and the dichloroacetate activated state [23].

### Biochemical Assays in Blood and Cerebrospinal fluid (CSF)

Complete blood cell counts, serum biochemistry profiles, urinalysis and CSF analysis were done at the VMTH. Pyruvate and lactate concentrations were measured in both CSF and plasma. Plasma samples were obtained at rest and following 10 minutes of strenuous exercise were collected and evaluated at the Comparative Neuromuscular Laboratory, School of Medicine, UC San Diego, as previously described [24].

### Pathology

Fresh tissue samples (skin, skeletal muscle and liver) were obtained either by surgical biopsy under general anesthesia or immediately after euthanasia. Muscle biopsy specimens were collected from the vastus lateralis and triceps brachii muscles and frozen immediately using isopentane precooled in liquid nitrogen. A standard panel of histochemical stains and reactions was performed on cryostat sections (10 μm thick) including HE, myofibrillar adenosine triphosphatase at pH 9.8, 4.5 and 4.3, modified Gomori trichrome, periodic acid-Schiff hematoxylin, esterase, staphylococcal protein A-horseradish peroxidase, oil red O, nicotinamide adenine dinucleotide tetrazolium reductase,and acid phosphatase as previously described [25].

Dogs with AHE euthanized at the VMTH had an immediate necropsy evaluation. The CNS and other issues were immersion-fixed in 10% formalin, and selected tissues were then routinely embedded in paraffin, sectioned at 5 μm and evaluated after HE staining. Selected brain sections were also histochemically stained with HE-Luxol fast blue. For transmission electron microscopy, skeletal muscle specimens were immersion fixed in 3% glutaraldehyde in buffer, routinely processed and embedded in plastic resin. Thick sections were stained with toluidine blue and appropriate thin sections selected for transmission electron microscopic evaluation as previously described [26].

### Molecular genetics techniques for candidate genes

Genomic DNA was isolated from cultured fibroblasts, blood or tissue using a Puregene genomic DNA isolation kit (Inter Medico, Markham, ON, Canada). RNA was isolated using Trizol (Life Technologies, Burlington, ON, Canada). Full length cDNA sequences were generated using RT-PCR and Superscript II reverse transcriptase and amplified using Platinum Hi-Fi Taq polymerase (Life Technologies, Burlington, ON, Canada). Oligonucleotide primers used for routine PCR (IDT, Iowa, USA) are listed in **Table** **5**. All products were sequenced by fluorescent sequencing methods as recommended (ACGT Corp., Toronto, ON, Canada).

**Table 5:** PCR primers for amplification of mtDNA and nuclear genes.

	Forward primer	Reverse primer
mtDNA (gDNA)		
MT-tRNA^LYS^, MT-ATP8, MT-ATP6	DogATP8F 5′-CTGATCTGCCTTAATAGTATAACCT-3′	DogATP6R 5′-GGTCATGGGCTTGGGTTG-3′
MT-tRNA^VAL^	Dog tRNAVal-F 5′-AAAACACAAGAGGAGACAAGTCG -3′	Dog tRNAVal-R 5′-CGGTACTATCTCTATCGCTCCAA-3′
MT-tRNA^LEU(UUR)^	DogtRNA-LeuF 5′-AACCTCCCCCAGTACGAAAG-3′	DogtRNA-LeuR 5′-AGGCTACGGCAAGAAGGATT-3′
MT-tRNA^SER(AGY)^	DogtRNA-Ser2F 5′-TGCCCCTACTCCTCCTATCC -3′	DogtRNA-Ser2R 5′-TCTGGAGTTGCACCAATTTTT-3′
MT-tRNA^TRY^, MT-tRNA^TYR^	DogtRNA-TrpF 5′-AAAAAGGCAACCCTATTACCC-3′	DogtRNA-TyrR 5′-GATGAGGAGGCTCAAAGCAG-3′
Nuclear genes (cDNA unless noted)		
*POLG* (4 parts)	DogPOLG-F 5′-CTTTCGGCCAGTAAAAGCAG-3′	POLG-R5 5′-AGTTCCCTCTGCCAAGCA-3′
	DogPOLG-F1 5′-GCGGCCAACTCGTTATTG-3′	DogPOLG-R1 5′-CCCCCATCTCCAACATGC-3′
	DogPOLG-F2 5′-GGACGTGTGGGCTACCTATG-3′	DogPOLG-R2 5′-ATGCCGCTCCGAGTAGTG-3′
	DogPOLG-F3 5′-CGGGTCACTCCAAAACTCAT-3′	DogPOLG-R3 5′-CCATACCACCATCTGGGAAC-3′
Twinkle	Dog-twinkle-F 5′-TAGTAAAGGCACCCGAACCA-3′	Dog-twinkle-R 5′-GCCTTAGCAGAGGGCTAAGAA-3′
TK2 (in two parts) (gDNA)	Dog-TK2-F 5′-GCCTTTAGGTGGATTGGACTG-3′	Dog-TK2-int1R 5′-CTGGGCCTTCTTTGACCTTA-3′
(cDNA)	DogTK2-ex3F 5′-ATCTGTGTTGAGGGCAATAT-3′	DogTK2-R2 5′-CTATGAACCATGTTTCTGATTCTCTG-3′
DGUOK	DogDGUOK-F 5′- AAATGTTCTCGGCGGAAGT-3′	DogDGUOK-R 5′-TGCAAAGTCGAAGACTAATACCA-3′
SUCLG1 (2 parts)	DogSUCLG1-F 5′-AATTCATTCAGGCGACTGCT-3′	DogSUCLG1-R1 5′-TTGATGATTCCAGGGCAGTT-3′
	DogSUCLG1-F1 5′-AGGACATGGTACGGGTCAAG-3′	DogSUCLG1-R 5′-CTTGCTGTACCGACAGACCA-3′
SUCLA2 (in two parts) (gDNA)	Dog-SUCLA2-F 5′-CATTTGATATTTGGCTGGAGGT-3′	Dog-SUCLA2-ex2R 5′-ATTCCTTTGTTGCTGCTGCT-3′
(cDNA)	Dog-SUCLA2-F3 5′-TTCTGGGAAGTTCTGGATTTTT-3′	Dog-SUCLA2-R1 5′-ATGCACAGCACAGTTCCATC-3′
MPV17 (3 parts) (gDNA)	DogMPV17-F4 5′-AGCCAAGCGCTCTTTAATTG-3′	DogMPV17int1R 5′-TGTGGTGAGGTGAGCTTCTG-3′
	DogMPV17int1F 5′-GGGACTTATTCCCTACCTGGA-3′	DogMPV17int4R 5′-ACCAAACCTGCCTTGTTCC-3′
	DogMPV17int4F 5′-GGTCTTTGAACTGGTCTGTGC-3′	DogMPV17int6R 5′-GCTGTGTCCAGCTGTTGTGA-3′
RRMB2	Dog-RRM2B-F 5′-CTCTGCCGGAGTTGGAGGT-3′	Dog-RRM2B-R 5′-TTCCCTAAGGAGGTGCTTTACA-3′
SLC19A3.1 (gDNA)	Exon 1 5′-CACCAGCCAGGGTTGTACTT-3′	5′-GGTTTAGCGCCTGCCTTT-3′
	Exon 2 5′-AGAAGGGGGAGGACCTCTTT-3′	5′-TTTCTTCCAGTGCCTTCCAT-3′
	Exon 3 5′-GCAAGTGACAGGGTTTATGGA-3′	5′-AAAAATCACAACCCGACAGTG-3′
	Exon 4 5′-TGGTGTTTTAATTCAGCCTTCA-3	5′-TATGGCAGGAGGAAAAGCAG-3′
	Exon 5 5′-TGGACCAGACCTGGAGATTC-3′	5′-CTGCTTTTCCTCCTGCCATA-3′
SLC19A3.2	5′-TTCTTGGGTTTTTCCCACAG-3′	5′-CTCTCCCAGGAGATCCCAGT-3′
SLC19A3	5′-AGCCCAGAGCACTACCAGAA-3′	5′-GGGCTCATCTGGATTCTGAC-3′
GAPDH	5′-AAGATTGTCAGCAATGCCTCC-3′	5′-CCAGGAAATGAGCTTGACAAA-3′

### Genome Wide Association

DNA extracted from blood samples from AHE and control dogs was genotyped using the Illumina HD canine array (Illumina Inc, San Diego, California). Association analysis was performed using PLINK software [27] (Shaun Purcell, URL: http://pngu.mgh.harvard.edu/purcell/plink/). Population stratification was evaluated by determining that the genomic inflation value was 1.0. SNPs with a minor allele frequency above 0.01 were used for the association analysis. Individuals with more than 15% missing calls were excluded from the analysis. SNPs with more than 10% missing genotypes were also excluded. 100,000 permutations were used to determine significance of associations. Genotypes were evaluated for homozygosity in affected individuals by visual inspection.

### Verification of *SLC19A3.1* Structure

To verify the structure of exon 2 in paralog *SLC19A3.1*, cDNA from a control sample was sequenced for this region and then compared to genomic sequence of canine genome assembly canfam 2.

### PCR and Sequencing of positional candidate gene SLC19A3

Each of the 5 exons of *SLC19A3.1* were amplified and sequenced in at least one dog with AHE and one control dog of a different breed. For areas of further interest, additional samples were sequenced from a dog with AHE, an unaffected AH, and an unaffected non-Alaskan Husky dog.

PCR was performed using primers that allowed amplification of all exons and intron/exon boundaries. Reactions were performed on an Applied Biosystems Gene Amp PCR System 9700. Each reaction consisted of 13.9 µl water, 2 µl 10X buffer with MgCl_2,_ 1 µl dNTP, 1 µl of each primer, 0.1 µl of DNA Taq Polymerase, and 1 µl of DNA. Cycling programs were based on the primers' Tm and the expected product size. Amplified samples were then sequenced on an Applied Biosystems 3100 Genetic Analyzer using the Big Dye Terminator Sequencing Kit. Sequences were aligned using VectorNTI software (Life Technologies, Burlington, ON, Canada).

### Genotyping

In order to screen a large number of normal control dogs, comprising both AH and other breed dogs, for the 4 bp insertion and SNP identified in exon 2, a PCR genotyping assay was developed using the following primers: 5′ 6FAM-ATCCTTGGCCTCTGTCTGTG, 3′-TAGGCATTGGGCTATTCACC. Genotyping was performed by fragment size on an Applied Biosystems 3100 Genetic Analyzer. Genotypes were analyzed using STRand software [28].

### RT-PCR

Semiquantitive RT-PCR was performed to compare the tissue expression of *SLC19A3.1* to that of *SLC19A3.2,* using cDNA made from 11 different tissues (spleen, skin, cerebellum, thymus, testis, spinal cord, heart, muscle, cerebral cortex, kidney, and liver) from one control dog (non-husky) sample. A reaction for the housekeeping gene GAPDH was also done to serve as a baseline to ensure equal concentrations and quality of the samples for expression comparison. RT-PCR was then performed using RNA extracted from both the cerebral cortex of an affected and an unaffected non-AH dog to directly compare expression of *SLC19A3.1* in the brain.
